The article "The Impact of Online Reviews on Consumers’ Purchasing Decisions: Evidence From an Eye-Tracking Study" was published in 2022. Journal: Front Psychol.

# The Impact of Online Reviews on Consumers’ Purchasing Decisions: Evidence From an Eye-Tracking Study

**DOI:** 10.3389/fpsyg.2022.865702

**Published:** 2022-06-08

**Authors:** Tao Chen, Premaratne Samaranayake, XiongYing Cen, Meng Qi, Yi-Chen Lan

**Affiliations:** ^1^School of Business, Ningbo University, Ningbo, China; ^2^School of Business, Western Sydney University, Penrith, NSW, Australia

**Keywords:** online reviews, eye-tracking, consumers purchasing decisions, emotion valence, gender

## Abstract

This study investigated the impact of online product reviews on consumers purchasing decisions by using eye-tracking. The research methodology involved (i) development of a conceptual framework of online product review and purchasing intention through the moderation role of gender and visual attention in comments, and (ii) empirical investigation into the region of interest (ROI) analysis of consumers fixation during the purchase decision process and behavioral analysis. The results showed that consumers’ attention to negative comments was significantly greater than that to positive comments, especially for female consumers. Furthermore, the study identified a significant correlation between the visual browsing behavior of consumers and their purchase intention. It also found that consumers were not able to identify false comments. The current study provides a deep understanding of the underlying mechanism of how online reviews influence shopping behavior, reveals the effect of gender on this effect for the first time and explains it from the perspective of attentional bias, which is essential for the theory of online consumer behavior. Specifically, the different effects of consumers’ attention to negative comments seem to be moderated through gender with female consumers’ attention to negative comments being significantly greater than to positive ones. These findings suggest that practitioners need to pay particular attention to negative comments and resolve them promptly through the customization of product/service information, taking into consideration consumer characteristics, including gender.

## Introduction

E-commerce has grown substantially over the past years and has become increasingly important in our daily life, especially under the influence of COVID-19 recently (Hasanat et al., 2020). In terms of online shopping, consumers are increasingly inclined to obtain product information from reviews. Compared with the official product information provided by the sellers, reviews are provided by other consumers who have already purchased the product *via* online shopping websites (Baek et al., 2012). Meanwhile, there is also an increasing trend for consumers to share their shopping experiences on the network platform (Floh et al., 2013). In response to these trends, a large number of studies (Floh et al., 2013; Lackermair et al., 2013; Kang et al., 2020; Chen and Ku, 2021) have investigated the effects of online reviews on purchasing intention. These studies have yielded strong evidence of the valence intensity of online reviews on purchasing intention. Lackermair et al. (2013), for example, showed that reviews and ratings are an important source of information for consumers. Similarly, through investigating the effects of review source and product type, Bae and Lee (2011) concluded that a review from an online community is the most credible for consumers seeking information about an established product. Since reviews are comments from consumers’ perspectives and often describe their experience using the product, it is easier for other consumers to accept them, thus assisting their decision-making process (Mudambi and Schuff, 2010).

The article "The Impact of Online Reviews on Consumers’ Purchasing Decisions: Evidence From an Eye-Tracking Study" was published in 2022. Journal: Front Psychol.

A survey conducted by Zhong-Gang et al. (2015) reveals that nearly 60% of consumers browse online product reviews at least once a week and 93% of whom believe that these online reviews help them to improve the accuracy of purchase decisions, reduce the risk of loss and affect their shopping options. When it comes to e-consumers in commercial activities on B2B and B2C platforms, 82% of the consumers read product reviews before making shopping choices, and 60% of them refer to comments every week. Research shows that 93% of consumers say online reviews will affect shopping choices, indicating that most consumers have the habit of reading online reviews regularly and rely on the comments for their purchasing decisions (Vimaladevi and Dhanabhakaym, 2012).

Consumer purchasing decision after reading online comments is a psychological process combining vision and information processing. As evident from the literature, much of the research has focused on the outcome and impact of online reviews affecting purchasing decisions but has shed less light on the underlying processes that influence customer perception (Sen and Lerman, 2007; Zhang et al., 2010; Racherla and Friske, 2013). While some studies have attempted to investigate the underlying processes, including how people are influenced by information around the product/service using online reviews, there is limited research on the psychological process and information processing involved in purchasing decisions. The eye-tracking method has become popular in exploring and interpreting consumer decisions making behavior and cognitive processing (Wang and Minor, 2008). However, there is very limited attention to how the emotional valence and the content of comments, especially those negative comments, influence consumers’ final decisions by adopting the eye-tracking method, including a gender comparison in consumption, and to whether consumers are suspicious of false comments.

The article "The Impact of Online Reviews on Consumers’ Purchasing Decisions: Evidence From an Eye-Tracking Study" was published in 2022. Journal: Front Psychol.

Thus, the main purpose of this research is to investigate the impact of online reviews on consumers’ purchasing decisions, from the perspective of information processing by employing the eye-tracking method. A comprehensive literature review on key themes including online reviews, the impact of online reviews on purchasing decisions, and underlying processes including the level and credibility of product review information, and processing speed/effectiveness to drive customer perceptions on online reviews, was used to identify current research gaps and establish the rationale for this research. This study simulated a network shopping scenario and conducted an eye movement experiment to capture how product reviews affect consumers purchasing behavior by collecting eye movement indicators and their behavioral datum, in order to determine whether the value of the fixation dwell time and fixation count for negative comment areas is greater than that for positive comment area and to what extent the consumers are suspicious about false comments. Visual attention by both fixation dwell time and count is considered as part of moderating effect on the relationship between the valence of comment and purchase intention, and as the basis for accommodating underlying processes.

The paper is organized as follows. The next section presents literature reviews of relevant themes, including the role of online reviews and the application of eye movement experiments in online consumer decision research. Then, the hypotheses based on the relevant theories are presented. The research methodology including data collection methods is presented subsequently. This is followed by the presentation of data analysis, results, and discussion of key findings. Finally, the impact of academic practical research and the direction of future research are discussed, respectively.

## Literature Review

### Online Product Review

Several studies have reported on the influence of online reviews, in particular on purchasing decisions in recent times (Zhang et al., 2014; Zhong-Gang et al., 2015; Ruiz-Mafe et al., 2018; Von Helversen et al., 2018; Guo et al., 2020; Kang et al., 2020; Wu et al., 2021). These studies have reported on various aspects of online reviews on consumers’ behavior, including consideration of textual factors (Ghose and Ipeirotiss, 2010), the effect of the level of detail in a product review, and the level of reviewer agreement with it on the credibility of a review, and consumers’ purchase intentions for search and experience products (Jiménez and Mendoza, 2013). For example, by means of text mining, Ghose and Ipeirotiss (2010) concluded that the use of product reviews is influenced by textual features, such as subjectivity, informality, readability, and linguistic accuracy. Likewise, Boardman and Mccormick (2021) found that consumer attention and behavior differ across web pages throughout the shopping journey depending on its content, function, and consumer’s goal. Furthermore, Guo et al. (2020) showed that pleasant online customer reviews lead to a higher purchase likelihood compared to unpleasant ones. They also found that perceived credibility and perceived diagnosticity have a significant influence on purchase decisions, but only in the context of unpleasant online customer reviews. These studies suggest that online product reviews will influence consumer behavior but the overall effect will be influenced by many factors.

The article "The Impact of Online Reviews on Consumers’ Purchasing Decisions: Evidence From an Eye-Tracking Study" was published in 2022. Journal: Front Psychol.

In addition, studies have considered broader online product information (OPI), comprising both online reviews and vendor-supplied product information (VSPI), and have reported on different attempts to understand the various ways in which OPI influences consumers. For example, Kang et al. (2020) showed that VSPI adoption affected online review adoption. Lately, Chen and Ku (2021) found a positive relationship between diversified online review websites as accelerators for online impulsive buying. Furthermore, some studies have reported on other aspects of online product reviews, including the impact of online reviews on product satisfaction (Changchit and Klaus, 2020), relative effects of review credibility, and review relevance on overall online product review impact (Mumuni et al., 2020), functions of reviewer’s gender, reputation and emotion on the credibility of negative online product reviews (Craciun and Moore, 2019) and influence of vendor cues like the brand reputation on purchasing intention (Kaur et al., 2017). Recently, an investigation into the impact of online review variance of new products on consumer adoption intentions showed that product newness and review variance interact to impinge on consumers’ adoption intentions (Wu et al., 2021). In particular, indulgent consumers tend to prefer incrementally new products (INPs) with high variance reviews while restrained consumers are more likely to adopt new products (RNPs) with low variance.

### Emotion Valence of Online Product Review and Purchase Intention

Although numerous studies have investigated factors that may influence the effects of online review on consumer behavior, few studies have focused on consumers’ perceptions, emotions, and cognition, such as perceived review helpfulness, ease of understanding, and perceived cognitive effort. This is because these studies are mainly based on traditional self-report-based methods, such as questionnaires, interviews, and so on, which are not well equipped to measure implicit emotion and cognitive factors objectively and accurately (Plassmann et al., 2015). However, emotional factors are also recognized as important in purchase intention. For example, a study on the usefulness of online film reviews showed that positive emotional tendencies, longer sentences, the degree of a mix of the greater different emotional tendencies, and distinct expressions in critics had a significant positive effect on online comments (Yuanyuan et al., 2009).

The article "The Impact of Online Reviews on Consumers’ Purchasing Decisions: Evidence From an Eye-Tracking Study" was published in 2022. Journal: Front Psychol.

Yu et al. (2010) also demonstrated that the different emotional tendencies expressed in film reviews have a significant impact on the actual box office. This means that consumer reviews contain both positive and negative emotions. Generally, positive comments tend to prompt consumers to generate emotional trust, increase confidence and trust in the product and have a strong persuasive effect. On the contrary, negative comments can reduce the generation of emotional trust and hinder consumers’ buying intentions (Archak et al., 2010). This can be explained by the rational behavior hypothesis, which holds that consumers will avoid risk in shopping as much as possible. Hence, when there is poor comment information presented, consumers tend to choose not to buy the product (Mayzlin and Chevalier, 2003). Furthermore, consumers generally believe that negative information is more valuable than positive information when making a judgment (Ahluwalia et al., 2000). For example, a single-star rating (criticism) tends to have a greater influence on consumers’ buying tendencies than that of a five-star rating (compliment), a phenomenon known as the negative deviation.

Since consumers can access and process information quickly through various means and consumers’ emotions influence product evaluation and purchasing intention, this research set out to investigate to what extent and how the emotional valence of online product review would influence their purchase intention. Therefore, the following hypothesis was proposed:

*H1*: For hedonic products, consumer purchase intention after viewing positive emotion reviews is higher than that of negative emotion ones; On the other hand, for utilitarian products, it is believed that negative comments are more useful than positive ones and have a greater impact on consumers purchase intention by and large.

The article "The Impact of Online Reviews on Consumers’ Purchasing Decisions: Evidence From an Eye-Tracking Study" was published in 2022. Journal: Front Psychol.

It is important to investigate Hypothesis one (H1) although it seems obvious. Many online merchants pay more attention to products with negative comments and make relevant improvements to them rather than those with positive comments. Goods with positive comments can promote online consumers’ purchase intention more than those with negative comments and will bring more profits to businesses.

Sen and Lerman (2007) found that compared with the utilitarian case, readers of negative hedonic product reviews are more likely to attribute the negative opinions expressed, to the reviewer’s internal (or non-product-related) reasons, and therefore, are less likely to find the negative reviews useful. However, in the utilitarian case, readers are more likely to attribute the reviewer’s negative opinions to external (or product-related) motivations, and therefore, find negative reviews more useful than positive reviews on average. Product type moderates the effect of review valence, Therefore, Hypothesis one is based on hedonic product types, such as fiction books.

Guo et al. (2020) found pleasant online customer reviews to lead to a higher purchase likelihood than unpleasant ones. This confirms hypothesis one from another side. The product selected in our experiment is a mobile phone, which is not only a utilitarian product but also a hedonic one. It can be used to make a phone call or watch videos, depending on the user’s demands.

### Eye-Tracking, Online Product Review, and Purchase Intention

The eye-tracking method is commonly used in cognitive psychology research. Many researchers are calling for the use of neurobiological, neurocognitive, and physiological approaches to advance information system research (Pavlou and Dimoka, 2010; Liu et al., 2011; Song et al., 2017). Several studies have been conducted to explore consumers’ online behavior by using eye-tracking. For example, using the eye-tracking method, Luan et al. (2016) found that when searching for products, customers’ attention to attribute-based evaluation is significantly longer than that of experience-based evaluation, while there is no significant difference for the experiential products. Moreover, their results indicated eye-tracking indexes, for example, fixation dwell time, could intuitively reflect consumers’ search behavior when they attend to the reviews. Also, Hong et al. (2017) confirmed that female consumers pay more attention to picture comments when they buy experience goods; when they buy searched products, they are more focused on the pure text comments. When the price and comment clues are consistent, consumers’ purchase rates significantly improve.

Eye-tracking method to explore and interpret consumers’ decision-making behavior and cognitive processing is primarily based on the eye-mind hypothesis proposed by Just and Carpenter (1992). Just and Carpenter (1992) stated that when an individual is looking, he or she is currently perceiving, thinking about, or attending to something, and his or her cognitive processing can be identified by tracking eye movement. Several studies on consumers’ decision-making behavior have adopted the eye-tracking approach to quantify consumers’ visual attention, from various perspectives including determining how specific visual features of the shopping website influenced their attitudes and reflected their cognitive processes (Renshaw et al., 2004), exploring gender differences in visual attention and shopping attitudes (Hwang and Lee, 2018), investigating how employing human brands affects consumers decision quality (Chae and Lee, 2013), consumer attention and different behavior depending on website content, functions and consumers goals (Boardman and McCormick, 2019). Measuring the attention to the website and time spent on each purchasing task in different product categories shows that shoppers attend to more areas of the website for purposes of website exploration than for performing purchase tasks. The most complex and time-consuming task for shoppers is the assessment of purchase options (Cortinas et al., 2019). Several studies have investigated fashion retail websites using the eye-tracking method and addressed various research questions, including how consumers interact with product presentation features and how consumers use smartphones for fashion shopping (Tupikovskaja-Omovie and Tyler, 2021). Yet, these studies considered users without consideration of user categories, particularly gender. Since this research is to explore consumers’ decision-making behavior and the effects of gender on visual attention, the eye-tracking approach was employed as part of the overall approach of this research project. Based on existing studies, it could be that consumers may pay more attention to negative evaluations, will experience cognitive conflict when there are contradictory false comments presented, and will be unable to judge good or bad (Cui et al., 2012). Therefore, the following hypothesis was proposed:

*H2*: Consumers’ purchasing intention associated with online reviews is moderated/influenced by the level of visual attention.

The article "The Impact of Online Reviews on Consumers’ Purchasing Decisions: Evidence From an Eye-Tracking Study" was published in 2022. Journal: Front Psychol.

To test the above hypothesis, the following two hypotheses were derived, taking into consideration positive and negative review comments from H1, and visual attention associated with fixation dwell time and fixation count.

*H2a*: When consumers intend to purchase a product, fixation dwell time and fixation count for negative comment areas are greater than those for positive comment areas.

Furthermore, when consumers browse fake comments, they are suspicious and actively seek out relevant information to identify the authenticity of the comments, which will result in more visual attention. Therefore, H2b was proposed:

*H2b*: Fixation dwell time and fixation count for fake comments are greater than those for authentic comments.

When considering the effect of gender on individual information processing, some differences were noted. For example, Meyers-Levy and Sternthal (1993) put forward the selectivity hypothesis, a theory of choice hypothesis, which implies that women gather all information possible, process it in an integrative manner, and make a comprehensive comparison before making a decision, while men tend to select only partial information to process and compare according to their existing knowledge—a heuristic and selective strategy. Furthermore, for an online product review, it was also reported that gender can easily lead consumers to different perceptions of the usefulness of online word-of-mouth. For example, Zhang et al. (2014) confirmed that a mixed comment has a mediating effect on the relationship between effective trust and purchasing decisions, which is stronger in women. This means that men and women may have different ways of processing information in the context of making purchasing decisions using online reviews. To test the above proposition, the following hypothesis was proposed:

*H3*: Gender factors have a significant impact on the indicators of fixation dwell time and fixation count on the area of interest (AOI). Male purchasing practices differ from those of female consumers. Male consumers’ attention to positive comments is greater than that of female ones, they are more likely than female consumers to make purchase decisions easily.

Furthermore, according to the eye-mind hypothesis, eye movements can reflect people’s cognitive processes during their decision process (Just and Carpenter, 1980). Moreover, neurocognitive studies have indicated that consumers’ cognitive processing can reflect the strategy of their purchase decision-making (Rosa, 2015; Yang, 2015). Hence, the focus on the degree of attention to different polarities and the specific content of comments can lead consumers to make different purchasing decisions. Based on the key aspects outlined and discussed above, the following hypothesis was proposed:

*H4*: Attention to consumers’ comments is positively correlated with consumers’ purchasing intentions: Consumers differ in the content of comments to which they gaze according to gender factors.

The article "The Impact of Online Reviews on Consumers’ Purchasing Decisions: Evidence From an Eye-Tracking Study" was published in 2022. Journal: Front Psychol.

Thus, the framework of the current study is shown in Figure 1.

**Figure 1:** Conceptual framework of the study.

## Materials and Methods

The research adopted an experimental approach using simulated lab environmental settings for collecting experimental data from a selected set of participants who have experience with online shopping. The setting of the task was based on guidelines for shopping provided on Taobao.com, which is the most famous and frequently used C2C platform in China. Each experiment was set with the guidelines provided and carried out for a set time. Both behavioral and eye movement data were collected during the experiment.

### Participants

A total of 40 healthy participants (20 males and 20 females) with online shopping experiences were selected to participate in the experiment. The participants were screened to ensure normal or correct-to-normal vision, no color blindness or poor color perception, or other eye diseases. All participants provided their written consent before the experiment started. The study was approved by the Internal Review Board of the Academy of Neuroeconomics and Neuromanagement at Ningbo University and by the Declaration of Helsinki (World Medical Association, 2014).

### Materials

With standardization and small selection differences among individuals, search products can be objectively evaluated and easily compared, to effectively control the influence of individual preferences on the experimental results (Huang et al., 2009). Therefore, this research focused on consumer electronics products, essential products in our life, as the experiment stimulus material. To be specific, as shown in Figure 2, a simulated shopping scenario was presented to participants, with a product presentation designed in a way that products are shown on Taobao.com. Figure 2 includes two segments: One shows mobile phone information (Figure 2A) and the other shows comments (Figure 2B). Commodity description information in Figure 2A was collected from product introductions on Taobao.com, mainly presenting some parameter information about the product, such as memory size, pixels, and screen size. There was little difference in these parameters, so quality was basically at the same level across smartphones. Prices and brand information were hidden to ensure that reviews were the sole factor influencing consumer decision-making. Product review areas in Figure 2B are the AOI, presented as a double-column layout. Each panel included 10 (positive or negative) reviews taken from real online shopping evaluations, amounting to a total of 20 reviews for each product. To eliminate the impact of different locations of comments on experimental results, the positions of the positive and negative comment areas were exchanged, namely, 50% of the subjects had positive comments presented on the left and negative comments on the right, with the remaining 50% of the participants receiving the opposite set up.

The article "The Impact of Online Reviews on Consumers’ Purchasing Decisions: Evidence From an Eye-Tracking Study" was published in 2022. Journal: Front Psychol.

**Figure 2:** Commodity information and reviews. **(A)** Commodity information, **(B)** Commodity reviews. Screenshots of Alibaba shopfront reproduced with permission of Alibaba and Shenzhen Genuine Mobile Phone Store.

A total of 12,403 product reviews were crawled through and extracted from the two most popular online shopping platforms in China (e.g., Taobao.com and JD.com) by using GooSeeker (2015), a web crawler tool. The retrieved reviews were then further processed. At first, brand-related, price-related, transaction-related, and prestige-related contents were removed from comments. Then, the reviews were classified in terms of appearance, memory, running speed, logistics, and so on into two categories: positive reviews and negative reviews. Furthermore, the content of the reviews was refined to retain the original intention but to meet the requirements of the experiment. In short, reviews were modified to ensure brevity, comprehensibility, and equal length, so as to avoid causing cognitive difficulties or ambiguities in semantic understanding. In the end, 80 comments were selected for the experiment: 40 positive and 40 negative reviews (one of the negative comments was a fictitious comment, formulated for the needs of the experiment). To increase the number of experiments and the accuracy of the statistical results, four sets of mobile phone products were set up. There were eight pairs of pictures in total.

### Procedures

Before the experiment started, subjects were asked to read the experimental guide including an overview of the experiment, an introduction of the basic requirements and precautions in the test, and details of two practice trials that were conducted. When participants were cognizant of the experimental scenario, the formal experiment was ready to begin. Participants were required to adjust their bodies to a comfortable sitting position. The 9 points correction program was used for calibration before the experiment. Only those with a deviation angle of less than 1-degree angle could enter the formal eye movement experiment. In our eye-tracking experiment, whether the participant wears glasses or not was identified as a key issue. If the optical power of the participant’s glasses exceeds 200 degrees, due to the reflective effect of the lens, the eye movement instrument will cause great errors in the recording of eye movements. In order to ensure the accuracy of the data recorded by the eye tracker, the experimenter needs to test the power of each participant’s glasses and ensure that the degree of the participant’s glasses does not exceed 200 degrees before the experiment. After drift correction of eye movements, the formal experiment began. The following prompt was presented on the screen: “you will browse four similar mobile phone products; please make your purchase decision for each mobile phone.” Participants then had 8,000 ms to browse the product information. Next, they were allowed to look at the comments image as long as required, after which they were asked to press any key on the keyboard and answer the question “are you willing to buy this cell phone?.”

The article "The Impact of Online Reviews on Consumers’ Purchasing Decisions: Evidence From an Eye-Tracking Study" was published in 2022. Journal: Front Psychol.

In this experiment, experimental materials were displayed on a 17-inch monitor with a resolution of 1,024 × 768 pixels. Participants’ eye movements were tracked and recorded by the Eyelink 1,000 desktop eye tracker which is a precise and accurate video-based eye tracker instrument, integrating with SR Research Experiment Builder, Data Viewer, and third-party software tools, with a sampling rate of 1,000 Hz. (Hwang and Lee, 2018). Data processing was conducted by the matching Data Viewer analysis tool.

The experiment flow of each trial is shown in Figure 3. Every subject was required to complete four trials, with mobile phone style information and comment content different and randomly presented in each trial. After the experiment, a brief interview was conducted to learn about participants’ browsing behavior when they purchased the phone and collected basic information *via* a matching questionnaire. The whole experiment took about 15 min.

**Figure 3:** Experimental flow diagram. Screenshots of Alibaba shopfront reproduced with permission of Alibaba and Shenzhen Genuine Mobile Phone Store.

### Data Analysis

Key measures of data collected from the eye-tracking experiment included fixation dwell time and fixation count. AOI is a focus area constructed according to experimental purposes and needs, where pertinent eye movement indicators are extracted. It can guarantee the precision of eye movement data, and successfully eliminate interference from other visual factors in the image. Product review areas are our AOIs, with positive comments (IA1) and negative comments (IA2) divided into two equal-sized rectangular areas.

Fixation can indicate the information acquisition process. Tracking eye fixation is the most efficient way to capture individual information from the external environment (Hwang and Lee, 2018). In this study, fixation dwell time and fixation count were used to indicate users’ cognitive activity and visual attention (Jacob and Karn, 2003). It can reflect the degree of digging into information and engaging in a specific situation. Generally, a more frequent fixation frequency indicates that the individual is more interested in the target resulting in the distribution of fixation points. Valuable and interesting comments attract users to pay more attention throughout the browsing process and focus on the AOIs for much longer. Since these two dependent variables (fixation dwell time and fixation count) comprised our measurement of the browsing process, comprehensive analysis can effectively measure consumers’ reactions to different review contents.

The article "The Impact of Online Reviews on Consumers’ Purchasing Decisions: Evidence From an Eye-Tracking Study" was published in 2022. Journal: Front Psychol.

## Results

The findings are presented in each section including descriptive statistical analysis, analysis from the perspective of gender and review type using ANOVA, correlation analysis of purchasing decisions, and qualitative analysis of observations.

### Descriptive Statistical Analysis

Fixation dwell time and fixation count were extracted in this study for each record. In this case, 160 valid data records were recorded from 40 participants. Each participant generated four records which corresponded to four combinations of two conditions (positive and negative) and two eye-tracking indices (fixation dwell time and fixation count). Each record represented a review comment. Table 1 shows pertinent means and standard deviations.

**Table 1:** Results of mean and standard deviations.

	Fixation dwell time (ms)				Fixation count			
	Positive review		Negative review		Positive review		Negative review	
	*M*	SD	*M*	SD	*M*	SD	*M*	SD
Male	10140.74	6048.38	11057.59	5236.95	45.76	25.91	49.1	20.83
Female	7262.06	4543.37	12334.06	7743.16	36.26	22.22	60.07	35.35
Total	8701.4	5524.34	11695.82	6620.13	41.01	24.53	54.59	29.44

It can be noted from the descriptive statistics for both fixation dwell time and fixation count that the mean of positive reviews was less than that of negative ones, suggesting that subjects spent more time on and had more interest in negative reviews. This tendency was more obvious in female subjects, indicating a role of gender.

Fixation results can be reported using a heat mapping plot to provide a more intuitive understanding. In a heat mapping plot, fixation data are displayed as different colors, which can manifest the degree of user fixation (Wang et al., 2014). Red represents the highest level of fixation, followed by yellow and then green, and areas without color represent no fixation count. Figure 4 implies that participants spent more time and cognitive effort on negative reviews than positive ones, as evidenced by the wider red areas in the negative reviews. However, in order to determine whether this difference is statistically significant or not, further inferential statistical analyses were required.

The article "The Impact of Online Reviews on Consumers’ Purchasing Decisions: Evidence From an Eye-Tracking Study" was published in 2022. Journal: Front Psychol.

**Figure 4:** Heat map of review picture.

### Repeated Measures From Gender and Review Type Perspectives—Analysis of Variance

The two independent variables for this experiment were the emotional tendency of the review and gender. A preliminary ANOVA analysis was performed, respectively, on fixation dwell time and fixation count values, with gender (man vs. woman) and review type (positive vs. negative) being the between-subjects independent variables in both cases.

A significant dominant effect of review type was found for both fixation dwell time (*p*_1_ < 0.001) and fixation count (*p*_2_ < 0.001; see Table 2). However, no significant dominant effect of gender was identified for either fixation dwell time (*p*_1_ = 0.234) or fixation count (*p*_2_ = 0.805). These results indicated that there were significant differences in eye movement indicators between positive and negative commentary areas, which confirms Hypothesis 2a. The interaction effect between gender and comment type was significant for both fixation dwell time (*p*_1_ = 0.002) and fixation count (*p*_2_ = 0.001). Therefore, a simple-effect analysis was carried out. The effects of different comment types with fixed gender factors and different gender with fixed comment type factors on those two dependent variables (fixation dwell time and fixation count) were investigated and the results are shown in Table 3.

**Table 2:** Results of ANOVA analysis.

	Fixation dwell time of AOI		Fixation count of AOI	
	*F*	Sig. (*p*_1_)	*F*	Sig. (*p*_2_)
Gender	1.42	0.234	0.061	0.805
Review type	19.842^*^	0.000	20.702^*^	0.000
Gender & Review type	9.552^*^	0.002	11.774^*^	0.001

* *Means significant when α = 0.05*.

**Table 3:** Results of simple-effect analysis.

Fixed factor	*I*	*J*	Fixation dwell time of AOI			Fixation count of AOI		
			Mean difference (I-J)	Standard error	Sig. (*p*_1_)	Mean difference (I-J)	Standard error	Sig. (*p*_2_)
Male	Positive reviews	Negative reviews	−916.85	950.68	0.336	−3.34	4.22	0.430
Female		
−5072.00^*^	950.68	0.000	−23.81^*^	4.22	0.000
Positive reviews	Male	Female	2878.66^*^	950.68	0.003	9.50^*^	4.22	0.025
Negative reviews			−1276.48	950.68	0.180	−10.98^*^	4.22	0.010

* *Means significant when α = 0.05*.

When the subject was female, comment type had a significant dominant effect for both fixation dwell time (*p*_1_ < 0.001) and fixation count (*p*_2_ < 0.001). This indicates that female users’ attention time and cognitive level on negative comments were greater than those on positive comments. However, the dominant effect of comment type was not significant (*p*_1_ = 0.336 > 0.05, *p*_2_ = 0.43 > 0.05) for men, suggesting no difference in concern about the two types of comments for men.

The article "The Impact of Online Reviews on Consumers’ Purchasing Decisions: Evidence From an Eye-Tracking Study" was published in 2022. Journal: Front Psychol.

Similarly, when scanning positive reviews, gender had a significant dominant effect (*p*_1_ = 0.003 < 0.05, *p*_2_ = 0.025 < 0.05) on both fixation dwell time and fixation count, indicating that men exerted longer focus and deeper cognitive efforts to dig out positive reviews than women. In addition, the results for fixation count showed that gender had significant dominant effects (*p*_1_ = 0.18 > 0.05, *p*_2_ = 0.01 < 0.05) when browsing negative reviews, suggesting that to some extent men pay significantly less cognitive attention to negative reviews than women, which is consistent with the conclusion that men’s attention to positive comments is greater than women’s. Although the dominant effect of gender was not significant (*p*_1_ = 0.234 > 0.05, *p*_2_ = 0.805 > 0.05) in repeated measures ANOVA, there was an interaction effect with review type. For a specific type of comment, gender had significant influences, because the eye movement index between men and women was different. Thus, gender plays a moderating role in the impact of comments on consumers purchasing behavior.

### Correlation Analysis of Purchase Decision

Integrating eye movement and behavioral data, whether participants’ focus on positive or negative reviews is linked to their final purchasing decisions were explored. Combined with the participants’ purchase decision results, the areas with large fixation dwell time and concerns of consumers in the picture were screened out. The frequency statistics are shown in Table 4.

**Table 4:** Frequency statistics of purchasing decisions.

		Whether to buy		Total
		No	Yes	
Review type (more attention)	Positive review	21	25	46
	Negative review	80	34	114
Total		101	59	160

The correlation analysis between the type of comment and the decision data shows that users’ attention level on positive and negative comments was significantly correlated with the purchase decision (*p* = 0.006 < 0.05). Thus, Hypothesis H4 is supported. As shown in Table 4 above, 114 records paid more attention to negative reviews, and 70% of the participants chose not to buy mobile phones. Also, in the 101 records of not buying, 80% of the subjects paid more attention to negative comments and chose not to buy mobile phones, while more than 50% of the subjects who were more interested in positive reviews chose to buy mobile phones. These experimental results are consistent with Hypothesis H1. They suggest that consumers purchasing decisions were based on the preliminary information they gathered and were concerned about, from which we can deduce customers’ final decision results from their visual behavior. Thus, the eye movement experiment analysis in this paper has practical significance.

The article "The Impact of Online Reviews on Consumers’ Purchasing Decisions: Evidence From an Eye-Tracking Study" was published in 2022. Journal: Front Psychol.

Furthermore, a significant correlation (*p* = 0.007 < 0.05) was found between the comments area attracting more interest and purchase decisions for women, while no significant correlation was found for men (*p* = 0.195 > 0.05). This finding is consistent with the previous conclusion that men’s attention to positive and negative comments is not significantly different. Similarly, this also explains the moderating effect of gender. This result can be explained further by the subsequent interview of each participant after the experiment was completed. It was noted from the interviews that most of the male subjects claimed that they were more concerned about the hardware parameters of the phone provided in the product information picture. Depending on whether it met expectations, their purchasing decisions were formed, and mobile phone reviews were taken as secondary references that could not completely change their minds.

Figure 5 shows an example of the relationship between visual behavior randomly selected from female participants and the correlative decision-making behavior. The English translation of words that appeared in Figure 5 is shown in Figure 4.

**Figure 5:** Fixation count distribution.

The subjects’ fixation dwell time and fixation count for negative reviews were significantly greater than those for positive ones. Focusing on the screen and running smoothly, the female participant decided not to purchase this product. This leads to the conclusion that this subject thought a lot about the phone screen quality and running speed while selecting a mobile phone. When other consumers expressed negative criticism about these features, the female participant tended to give up buying them.

Furthermore, combined with the result of each subject’s gaze distribution map and AOI heat map, it was found that different subjects paid attention to different features of mobile phones. Subjects all had clear concerns about some features of the product. The top five mobile phone features that subjects were concerned about are listed in Table 5. Contrary to expectations, factors, such as appearance and logistics, were no longer a priority. Consequently, the reasons why participants chose to buy or not to buy mobile phones can be inferred from the gazing distribution map recorded in the product review picture. Therefore we can provide suggestions on how to improve the design of mobile phone products for businesses according to the features that users are more concerned about.

**Table 5:** Top 5 features of mobile phones.

**Top**	1	2	3	4	5
**Features**	Running smoothly	Battery life	Fever condition	Pixel	After-sale service

The article "The Impact of Online Reviews on Consumers’ Purchasing Decisions: Evidence From an Eye-Tracking Study" was published in 2022. Journal: Front Psychol.

### Fictitious Comments Recognition Analysis

The authenticity of reviews is an important factor affecting the helpfulness of online reviews. To enhance the reputation and ratings of online stores, in the Chinese e-commerce market, more and more sellers are employing a network “water army”—a group of people who praise the shop and add many fake comments without buying any goods from the store. Combined with online comments, eye movement fixation, and information extraction theory, Song et al. (2017) found that fake praise significantly affects consumers’ judgment of the authenticity of reviews, thereby affecting consumers’ purchase intention. These fictitious comments glutted in the purchasers’ real ones are easy to mislead customers. Hence, this experiment was designed to randomly insert a fictitious comment into the remaining 79 real comments without notifying the participants in advance, to test whether potential buyers could identify the false comments and find out their impact on consumers’ purchase decisions.

The analysis of the eye movement data from 40 product review pictures containing this false commentary found that only several subjects’ visual trajectories were back and forth in this comment, and most participants exhibited no differences relative to other comments, indicating that the vast majority of users did not identify the lack of authenticity of this comment. Moreover, when asked whether they had taken note of this hidden false comment in interviews, almost 96% of the participants answered they had not. Thus, Hypothesis H2b is not supported.

This result explains why network “water armies” are so popular in China, as the consumer cannot distinguish false comments. Thus, it is necessary to standardize the e-commerce market, establish an online comment authenticity automatic identification information system, and crack down on illegal acts of employing network troops to disseminate fraudulent information.

## Discussion and Conclusion

In the e-commerce market, online comments facilitate online shopping for consumers; in turn, consumers are increasingly dependent on review information to judge the quality of products and make a buying decision. Consequently, studies on the influence of online reviews on consumers’ behavior have important theoretical significance and practical implications. Using traditional empirical methodologies, such as self-report surveys, it is difficult to elucidate the effects of some variables, such as review choosing preference because they are associated with automatic or subconscious cognitive processing. In this paper, the eye-tracking experiment as a methodology was employed to test congruity hypotheses of product reviews and explore consumers’ online review search behavior by incorporating the moderating effect of gender.

The article "The Impact of Online Reviews on Consumers’ Purchasing Decisions: Evidence From an Eye-Tracking Study" was published in 2022. Journal: Front Psychol.

Hypotheses testing results indicate that the emotional valence of online reviews has a significant influence on fixation dwell time and fixation count of AOI, suggesting that consumers exert more cognitive attention and effort on negative reviews than on positive ones. This finding is consistent with Ahluwalia et al.’s (2000) observation that negative information is more valuable than positive information when making a judgment. Specifically, consumers use comments from other users to avoid possible risks from information asymmetry (Hong et al., 2017) due to the untouchability of online shopping. These findings provide the information processing evidence that customers are inclined to acquire more information for deeper thinking and to make a comparison when negative comments appear which could more likely result in choosing not to buy the product to reduce their risk. In addition, in real online shopping, consumers are accustomed to giving positive reviews as long as any dissatisfaction in the shopping process is within their tolerance limits. Furthermore, some e-sellers may be forging fake praise (Wu et al., 2020). The above two phenomena exaggerate the word-of-mouth effect of negative comments, resulting in their greater effect in contrast to positive reviews; hence, consumers pay more attention to negative reviews. Thus, Hypothesis H2a is supported. However, when limited fake criticism was mixed in with a large amount of normal commentary, the subject’s eye movements did not change significantly, indicating that little cognitive conflict was produced. Consumers could not identify fake comments. Therefore, H2b is not supported.

Although the dominant effect of gender was not significant on the indicators of the fixation dwell time and fixation count, a significant interaction effect between user gender and review polarity was observed, suggesting that consumers’ gender can regulate their comment-browsing behavior. Therefore, H3 is partly supported. For female consumers, attention to negative comments was significantly greater than positive ones. Men’s attention was more homogeneous, and men paid more attention to positive comments than women. This is attributed to the fact that men and women have different risk perceptions of online shopping (Garbarino and Strahilevitz, 2004). As reported in previous studies, men tend to focus more on specific, concrete information, such as the technical features of mobile phones, as the basis for their purchase decision. They have a weaker perception of the risks of online shopping than women. Women would be worried more about the various shopping risks and be more easily affected by others’ evaluations. Specifically, women considered all aspects of the available information, including the attributes of the product itself and other post-use evaluations. They tended to believe that the more comprehensive the information they considered, the lower the risk they faced of a failed purchase (Garbarino and Strahilevitz, 2004; Kanungo and Jain, 2012). Therefore, women hope to reduce the risk of loss by drawing on as much overall information as possible because they are more likely to focus on negative reviews.

The article "The Impact of Online Reviews on Consumers’ Purchasing Decisions: Evidence From an Eye-Tracking Study" was published in 2022. Journal: Front Psychol.

The main finding from the fixation count distribution is that consumers’ visual attention is mainly focused on reviews containing the following five mobile phone characteristics: running smoothly, battery life, fever condition of phones, pixels, and after-sales service. Considering the behavior results, when they pay more attention to negative comments, consumers tend to give up buying mobile phones. When they pay more attention to positive comments, consumers often choose to buy. Consequently, there is a significant correlation between visual attention and behavioral decision results. Thus, H4 is supported. Consumers’ decision-making intention can be reflected in the visual browsing process. In brief, the results of the eye movement experiment can be used as a basis for sellers not only to formulate marketing strategies but also to prove the feasibility and strictness of applying the eye movement tracking method to the study of consumer decision-making behavior.

### Theoretical Implications

This study has focused on how online reviews affect consumer purchasing decisions by employing eye-tracking. The results contribute to the literature on consumer behavior and provide practical implications for the development of e-business markets. This study has several theoretical contributions. Firstly, it contributes to the literature related to online review valence in online shopping by tracking the visual information acquisition process underlying consumers’ purchase decisions. Although several studies have been conducted to examine the effect of online review valence, very limited research has been conducted to investigate the underlying mechanisms. Our study advances this research area by proposing visual processing models of reviews information. The findings provide useful information and guidelines on the underlying mechanism of how online reviews influence consumers’ online shopping behavior, which is essential for the theory of online consumer behavior.

The article "The Impact of Online Reviews on Consumers’ Purchasing Decisions: Evidence From an Eye-Tracking Study" was published in 2022. Journal: Front Psychol.

Secondly, the current study offers a deeper understanding of the relationships between online review valence and gender difference by uncovering the moderating role of gender. Although previous studies have found the effect of review valence on online consumer behavior, the current study first reveals the effect of gender on this effect and explains it from the perspective of attention bias.

Finally, the current study investigated the effect of online reviews on consumer behavior from both eye-tracking and behavioral self-reports, the results are consistent with each other, which increased the credibility of the current results and also provides strong evidence of whether and how online reviews influence consumer behavior.

### Implications for Practice

This study also has implications for practice. According to the analysis of experimental results and findings presented above, it is recommended that online merchants should pay particular attention to negative comments and resolve them promptly through careful analysis of negative comments and customization of product information according to consumer characteristics including gender factors. Based on the findings that consumers cannot identify false comments, it is very important to establish an online review screening system that could automatically screen untrue content in product reviews, and create a safer, reliable, and better online shopping environment for consumers.

### Limitations and Future Research

Although the research makes some contributions to both theoretical and empirical literature, it still has some limitations. In the case of experiments, the number of positive and negative reviews of each mobile phone was limited to 10 positive and 10 negative reviews (20 in total) due to the size restrictions on the product review picture. The number of comments could be considered relatively small. Efforts should be made in the future to develop a dynamic experimental design where participants can flip the page automatically to increase the number of comments. Also, the research was conducted to study the impact of reviews on consumers’ purchase decisions by hiding the brand of the products. The results would be different if the brand of the products is exposed since consumers might be moderated through brand preferences and brand loyalty, which could be taken into account in future research projects.

## Data Availability Statement

The original contributions presented in the study are included in the article/supplementary material, further inquiries can be directed to the corresponding author.

## Author Contributions

TC conceived and designed this study. TC, PS, and MQ wrote the first draft of the manuscript. TC, XC, and MQ designed and performed related experiments, material preparation, data collection, and analysis. TC, PS, XC, and Y-CL revised the manuscript. All authors contributed to the article and approved the submitted version.

The article "The Impact of Online Reviews on Consumers’ Purchasing Decisions: Evidence From an Eye-Tracking Study" was published in 2022. Journal: Front Psychol.

## Conflict of Interest

The authors declare that the research was conducted in the absence of any commercial or financial relationships that could be construed as a potential conflict of interest.

## Publisher’s Note

All claims expressed in this article are solely those of the authors and do not necessarily represent those of their affiliated organizations, or those of the publisher, the editors and the reviewers. Any product that may be evaluated in this article, or claim that may be made by its manufacturer, is not guaranteed or endorsed by the publisher.
